This article has been retracted.

# Digital inclusive finance, R&D investment, and green technology innovation nexus

**DOI:** 10.1371/journal.pone.0297264

**Published:** 2024-01-19

**Authors:** Hongying Sun, Yipei Luo, Jia Liu, Miraj Ahmed Bhuiyan

**Affiliations:** School of Economics, Guangdong University of Finance and Economics, Guangzhou, China; University of Galway, Ireland / Anhui University of Finance and Economics, CHINA

## Abstract

Green technology innovation is an effective means to achieve high-quality economic development. The impact and mechanism of digital financial inclusion on regional green technology innovation are tested using a threshold regression model and the panel fixed effect model, based on China’s provincial Panel data (provincial Panel data are regional annual report data) from 2011 to 2020. According to the study, there is a direct link between local green technology innovation and digital financial inclusion. This paper highlights the differences in their influence by location and usage depth and underscores the necessity of government engagement to improve these characteristics. Information infrastructure needs to be strengthened, especially in areas with gaps. Greater investment in research and development (R&D) indirectly supports regional green technology innovation since it is impacted by digital financial inclusion. Interestingly, a threshold effect becomes most noticeable when digital financial inclusion rises above a particular threshold. Promoting utilizing digital financial inclusion to lessen regional differences in green technology innovation is important.

## 1. Introduction

Under the superimposed development of industrialization, informatization, and modernization, green technology innovation has gradually become an essential branch of the new round of the global industrial revolution and scientific and technological competition. Chinese-style green modernization requires establishing and improving a green and low-carbon circular development economic system, creating a driving force with green technology innovation as the core [1], and comprehensively promoting high-quality development and high-level protection. On the one hand, guiding the market-oriented development of green technology innovation is conducive to enhancing the decisive role of the market in resource allocation and innovation connection, stimulating the vitality of various innovative entities, and fully attracting diversified capital to settle in the green field. On the other hand, it is also conducive to promoting intelligent equipment, industrial ecology, and improving international environmental leadership.

Considering the existence of financing constraints, green technology innovation is inseparable from the support of a sound financial system. The financial exclusion phenomenon has become increasingly intense in this field and has gradually become the bottleneck in developing green technology innovation. The main reasons include: First, the long cycle of transforming green technology innovation results in increased financial pressure and achievement of transformation risks, directly leading to investors’ hesitation. Second, the capacity and inadequacy of information disclosure of green technology innovation inputs and outputs have exacerbated information asymmetry, resulting in transaction costs reducing financial market effectiveness [2]. Thus, lenders’ control of corporate risk and credit has decreased [3], and financial institutions have become increasingly conservative in allocating capital to green technology innovation. Third, the growing profit-seeking incentives of financial institutions mismatch their risk appetite with the growing needs of the green technology innovation industry [4]. Inclusive financial services have emerged with the rapid promotion and deepening application of information technologies such as the Internet, big data, and cloud computing in the financial field [5]. Based on the requirements of equal opportunities and the principle of business sustainability, it meets the financial needs of all levels and groups of society at an affordable cost, and its breadth and depth have been further expanded. Digital Inclusive Finance optimized with the help of digital technology has greatly reduced the cost of inclusive financial services and effectively solved the contradiction of Financial Exclusion, which has received great attention from academia and practice [6].

Relying on the platforms of banks, non-bank financial institutions, and financial technology enterprises, digital Inclusive Finance provides more comprehensive and high-quality financial services for small and micro enterprises, farmers, and low-income groups by combining traditional finance and digital technology. It creates favorable conditions for the innovative development of enterprises and regions with its advantages of wide coverage, low cost, and high efficiency. The existing literature shows that digital Inclusive Finance incentivizes enterprise and regional innovation [7, 8]. The allocation of credit resources, regional consumption quality, population education level, and infrastructure construction [9] are important transmission mechanisms.

Based on this, this article will deeply analyze the impact of the relationship between digital finance and green technology innovation from theoretical and empirical perspectives. This will help fully understand the current quality of green development in China and provide policy recommendations.

## 2. Literature review

The relevant literature on digital Financial inclusion, R&D investment, and green technology innovation can be divided into three aspects. First, research on digital Financial inclusion and R&D investment. For example, Meng et al. [10] found that developing digital Financial inclusion and its coverage, depth of use, and digitalization of its three sub-dimensions significantly promote enterprise R&D investment by building a two-way fixed effect model. Zhu [11] found that the improvement of digital financial inclusion plays a stronger role in promoting the level of R&D investment intensity of enterprises by using the data of A-share listed companies from 2011 to 2020. Second, research on digital Financial inclusion and green technology innovation. For example, Zhang [12] found that the development of digital Financial inclusion and its coverage, depth of use, and digitalization of its three sub-dimensions significantly promote regional innovation capability by building a fixed effect model and threshold model. A recent study by Xu et al. [13] concludes that enthusiasm has less impact on the quality of green technology innovation than the development of Digital inclusive finance. Yin [14] also found that digital Financial inclusion has a positive role in promoting the efficiency of green technology innovation by building a spatial Durbin econometric model. Lin [15] also supports the idea that digital finance can improve the quantity and quality of green technological innovation. Xu [16] found by building the spatial panel model and threshold panel model that digital Financial inclusion not only has a significant positive effect on the innovation ability of the region but also its spillover effect will drive the improvement of the innovation ability of surrounding regions. The third is research on R&D investment and green technology innovation. Xu et al. [17] used the system dynamics method to analyze the impact of government R&D investment on enterprise R&D investment. They found that government R&D investment has a dual effect of leverage and crowding out on enterprise R&D investment, with an inverted U-shaped relationship between them. Romer [18] believes that R&D investment can significantly improve innovation efficiency and promote economic growth through technological progress and was the first to analyze the positive effect of government investment in enterprise R&D on economic growth. Park [19] used an improved Romer model by simultaneously introducing government R&D investment and enterprise R&D investment. The study found that government R&D investment indirectly improves economic development, while enterprise R&D investment directly promotes economic growth.

Digital Inclusive Finance not only promotes economic development but can effectively suppress the ecological footprint [20] and carbon productivity [21] and achieve sustainable development goals [22]. Razzaq [23] also indicates that the marginal contribution of digital green finance towards green growth is substantial. Cao [24] pointed out that digital finance significantly improves energy-environmental performance in China.

To sum up, many studies focus on the relationship between digital Financial inclusion, R&D investment, and green technology innovation development but less on the relationship between the three under a unified analytical framework. In particular, the impact of digital Financial inclusion on R&D investment is not yet clear. At the same time, only considering the impact of digital Financial inclusion on green technological innovation or the impact of R&D investment on technological innovation cannot fully reflect the dynamic relationship within the system. According to relevant literature research, digital Financial inclusion has a significant role in promoting R&D investment, and R&D investment will also directly or indirectly promote regional green technology innovation. Therefore, this paper explores the relationship among digital Financial inclusion, R&D investment, and green technology innovation by building a Mesomeric effect model. First, based on the digital Financial inclusion index of Peking University, taking the Panel data of provinces and cities across the country from 2011 to 2020 as the sample, analyze the relationship between digital Financial inclusion and green technology innovation. The second is to divide the region into the southern and northern regions according to economic geography and analyze the regional heterogeneity of digital Financial inclusion on green technology innovation. Third, through the Mesomeric effect, the impact of industrial structure upgrading on digital Financial inclusion and green technology innovation is analyzed in depth. The fourth is to explore the nonlinear characteristics of digital Financial inclusion in green technology innovation through a threshold regression model.

## 3. Theoretical analysis

Green technology innovation refers to improving existing production processes, methods, services, and business models by enterprises to use resources more efficiently and in an environmentally friendly manner to achieve the purpose of positive externalities on the environment. As an important extension and application of the digital economy, inclusive digital finance has introduced digital technology to the traditional financial field, mainly through the following channels to promote the development of green technology innovation.

### 3.1 The direct mechanism of digital inclusive finance and green technology innovation

Digital Financial inclusion can use Big data, blockchain, and other technologies to solve the problems enterprises face in green innovation, such as slow market returns, low fault tolerance rates, and large working capital investments. On the one hand, as an important part of the Financial inclusion system, digital Financial inclusion can not only reduce the threshold of financial services [25], improve the efficiency of enterprise financing [26] but also reduce the cost of enterprise financing [27], effectively easing the financing constraints of enterprises. On the other hand, digital Financial inclusion can use the Internet and other technologies to break the restrictions of time, space, and workforce, significantly reduce the transaction cost and time cost of enterprise financing [28], reduce the cost of innovation, and promote green technology innovation. At the same time, digital Financial inclusion can establish a dynamic and effective risk control system through digital technology, improve risk identification ability, effectively evaluate project risk information, and improve credit suppliers’ risk control level. In addition, digital Financial inclusion can also launch special green credit for green projects and use policy preferences to allow funds to flow to green innovation more efficiently. Therefore, digital Financial inclusion can provide more efficient financing models, lower financing costs for green enterprises and projects, and promote green technology innovation [29]. Based on this, this article proposes hypothesis 1.

*Hypothesis 1*: *The development of digital Financial inclusion promotes green technology innovation*.

### 3.2 The indirect mechanism of inclusive digital finance on green technology innovation

With the support of inclusive digital finance, green enterprises can form credit and effectively broaden the financing channels for green technology innovation [30]. It is conducive to enterprises, institutions, universities, and other R & D entities to obtain more R & D funds, ease financing constraints, and improve R & D investment in enterprises [31]. There are two primary sources of corporate credit: operating cash flow and third-party guarantees [32]. The operational cash flow reflects the enterprise’s financial information, operating information, market position, and product advantages. These are all critical bases for the supply of funds, such as commercial banks, to judge whether the innovative project can be repaid on time and whether the green innovation project is an investment- and the key to forming green enterprise credit. The funding provider quickly integrates actual enterprise data through cloud computing, big data, and blockchain technologies. It can analyze and predict the future cash flow of green technology projects, alleviate the contradiction of information asymmetry to a certain extent, and solve the financing difficulties of R&D entities due to credit qualifications, scale levels, and other reasons [33].

The increase in the intensity of R&D investment can promote green technology innovation. R&D Investment is a resource allocation for technological innovation, including talent, capital, knowledge, and other investment elements. According to endogenous growth theory and human capital theory, human capital, knowledge spillover, and capital accumulation are all-important development factors to promote technological innovation [34]. At the same time, capital investment promotes technological innovation better than human capital, so Digital Inclusive Finance can effectively promote technological innovation by increasing investment in R&D capital [35].

*Hypothesis 2*: *Digital financial inclusion promotes green technology innovation by increasing investment in research and development*.

### 3.3 The nonlinear transmission mechanism of inclusive digital finance to green technology innovation

Digital Financial inclusion integrates traditional finance and digital technology (such as Big data, blockchain, Internet, and 5G) to provide more comprehensive and high-quality financial services [36]. First, the cost of digital financial inclusion was high initially, and the integration of digital technology and traditional finance was low. Not only was the investment in digital infrastructure huge, but also the green finance business structure was single, and the available data was limited, resulting in low prediction and analysis ability, low technology spillover effect, and ultimately, the promotion of digital Financial inclusion on green technology innovation was weak. With the development of digital Financial inclusion businesses and the support of green policies, green environmental protection has taken root. Digital Financial inclusion can promote green technology innovation by improving the efficiency of financial resource allocation [37]. Secondly, digital Financial inclusion naturally carries multiple elements such as informatization, networking, and intelligence [38], which will inevitably affect green innovation through new-generation information technologies like the Internet. In empowering digital finance, as the participation of green innovation entities continues to increase, the inherent value of digital financial services begins to exhibit nonlinear geometric growth. As digital finance improves, its empowering effect on green innovation may increase by leaps and bounds [39]. As digital finance empowers green innovation to enter the deep water zone, more green innovation entities can fully enjoy the spillover dividends of green innovation on a larger scale at lower costs. At a higher efficiency level, leading to a continuous strengthening of the empowering effect of digital finance on green innovation, there is a significant "network effect" (network effect refers to the jumping increase of its impact with the rise in internet usage scale within a specific range). Therefore, digital Financial inclusion may play different roles in promoting green technology at different stages of development. Thus, this paper proposes Hypothesis 3. However, Fig 1 shows the mechanism diagram of the impact of Digital Inclusive Finance on green technology innovation.

**Fig 1:** Mechanism diagram of the impact of digital inclusive finance on green technology innovation.

*Hypothesis 3*: *The role of digital financial inclusion in promoting enterprises’ green technology innovation shows a nonlinear characteristic*.

## 4. The selection of indicators and model design

### 4.1 Variable selection

**i) Explained variable- green technology innovation (GTP)**
  The research evaluation of green technology innovation mainly adopts the number of green invention patents, including the number of applications and grants. Because technological innovation is the embodiment of resource input and uses efficiency, the number of patents representing innovation output can better reflect the innovation ability of the region. It is generally believed that the innovation of patents from high to low is invention patents, utility model patents, and design patents, which means that invention patents have the highest gold content. Therefore, we can choose the number of green invention patents granted Gtp1 and the number of green invention patents declared Gtp2 to evaluate green technology innovation in different regions in China. At the same time, the ratio of green invention patent authorization to all patents in the current year, Gtp3, is used to replace the explanatory variable for the robustness test. Among them, the number of green invention patents granted is based on the International Patent Classification (IPC) code of green patents issued by the Global Intellectual Property Office (WIPO) and then summarized according to the patent application data submitted by the State Intellectual Property Office.
**ii) Explanatory variables; Digital finance (Inf).** In this paper, the second issue of the "Peking University Digital Inclusive Finance Index," jointly compiled by the Digital Finance Research Center of Peking University and Ant Financial, is selected as the proxy variable for the development level of digital Finance (Guo, 2020). At the same time, the two levels of Digital Inclusive Finance, the breadth of use and the depth of application are expressed in *Inf_di* and *Inf _de*, respectively.
**iii) Mediation variables- R&D investment (R&D).** Capital investment is an important supporting factor in the innovation process. This paper selects the proportion of internal expenditure on research and experimental development in each region to the regional GDP as an R&D input indicator [40].
**iv) Control variables.** To ensure the robustness of the results, this paper adopts the following control variables: (1) the level of traditional financial development (Tf): the balance of loans of financial institutions/GDP [41]. (2) the degree of fiscal decentralization (Finadp): the revenue ratio within the fiscal budget to the fiscal budget. (3) Human capital level (HC): This paper draws on the method of Li et al. [42] and adopts the actual per capita human capital level of each province published by the China Human Capital and Labor Economics Research Center of the Central University of Finance and Economics as a proxy variable for the regional human capital level. For the specific calculation method of this indicator, please refer to the "China Human Capital Report (2019)". (4) Institutional quality (Mi): Drawing on previous research, this paper uses the regional marketization index as a proxy variable for institutional quality. The data comes from the "Marketization Index Report by Provinces in China (2018)" compiled by [43]. China’s marketization index reflects the degree of marketization in China from five levels: legal and regulatory system environment, industrial market development, government policy and market, non-state-owned economy development, and marketization of scientific and technological achievements. It not only fully reflects China’s marketization level in various fields but is also the most widely used index by the international academic community to judge the quality of China’s regional institutions. (5) Level of economic development (*Lnpgdp*): expressed by the logarithm of *GDP* per capita.

### 4.2 Model establishment

First of all, to study the direct impact of inclusive digital finance on green technology innovation, this paper is interpreted by the variable green technology innovation measured by the number of green patents granted Gtp 1 and the number of declarations G*tp*2, and the following panel fixed regression model is set up:

$$Gtp_{it}=\alpha_{0}+\alpha_{1}Inf_{it}+\delta control_{it}+v_{i}+\mu_{t}+\varepsilon_{it}$$ (1)

In Eq (1), *i* stands for an individual; *t* represents the year; *control*_*it*_ Represents a control variable; *v*_*i*_ Represents individual effects; *μ*_*t*_ Represents a time effect; *ε*_*it*_ represents a random disturbance term.

Subsequently, the following model is established to verify whether R&D investment intensity plays an intermediary role in the impact mechanism of Digital Inclusive Finance on green technology innovation:

$${R\&D}_{i,t}=\gamma_{0}+\gamma_{1}\mathrm{In}f_{it}+\lambda {\mathrm{control}}_{it}+v_{i}+\mu_{t}+\varepsilon_{it}$$ (2)

$$Gtp1_{it}=\delta_{0}+\delta_{1}\mathrm{In}f_{it}+\delta_{2}{R\&D}_{i,t}+\lambda {\mathrm{control}}_{it}+v_{i}+\mu_{t}+\varepsilon_{it}$$ (3)

$$Gtp2_{it}=\delta_{0}+\delta_{1}\mathrm{In}f_{it}+\delta_{2}{R\&D}_{i,t}+\lambda {\mathrm{control}}_{it}+v_{i}+\mu_{t}+\varepsilon_{it}$$ (4)

Finally, the impact of different levels of digital inclusive finance development on green technology innovation may be nonlinear, so a panel threshold model is established to study the nonlinear mechanism of inclusive digital finance on green technology innovation:

$$Gt{p1}_{it}=\alpha_{0}+\alpha_{1}\mathrm{In}f_{it}\cdot I(\mathrm{In}f_{it}\leq Z_{1})+\alpha_{2}\mathrm{In}f_{it}\cdot I(Z_{1}<\mathrm{In}f_{it}\leq Z_{2})+\alpha_{3}\mathrm{In}f_{it}\cdot I(\ln df_{it}>Z_{2})+\lambda {\mathrm{control}}_{it}+v_{i}+\mu_{t}+\varepsilon_{it}$$ (5)

where: *Z*_1_, *Z*_2_ is the threshold for digital finance, *I*() is an indicator function. The other variables are interpreted as above.

### 4.3 Data sources and descriptive statistics

This paper uses 30 provinces, municipalities, and autonomous regions across China from 2011 to 2021 (Due to the lack of data in Hong Kong, Macao, Taiwan, and the Tibet Autonomous Region, this article is not considered in this article) as a research sample. The data are from the China Digital Inclusive Finance Index, the National Bureau of Statistics, and the China Statistical Yearbook released by the Digital Finance Research Center of Peking University. The missing values are supplemented by linear interpolation. The descriptive statistical results of each variable are shown in Table 1. To make the final result not affected by the data dimension, all variables are standardized in this paper. Michal and Daniel [44] put them into the regression equation, and the above continuous variables are subject to up and down 1% tailing.

**Table 1:** Descriptive statistics for variables.

	Variable symbols	Variable name	Sample size	mean	standard deviation	Minimum value	Maximum value
Interpreted variables	*Gtp*1	Number of green invention patents authorized	300	964.6	1355	5	7412
	*Gtp*2	Number of green invention patent applications	300	4180	6053	15	31391
	*Gtp*3	The number of green invention patents granted accounts for the proportion of all patents	300	0.0190	0.00980	0.00470	0.0658
Explanatory variables	*Inf*	Digital Inclusive Finance	300	217.2	96.97	18.33	431.9
	*Inf_di*	Use the breadth index	300	290.2	117.6	7.580	462.2
	*Inf _de*	Use the depth index	300	212.0	98.11	6.760	488.7
Mediation variables	*R&D* input	R&D investment	300	0.0174	0.0112	0.00420	0.0647
Control variables	*Tf*	The level of traditional financial development	300	1.570	1.014	0.195	6.636
	*Finadp*	Fiscal decentralization	300	0.497	0.190	0.151	0.931
	*Mi*	Market-oriented index	300	6.706	1.919	2.372	11.11
	*Hc*	The level of human capital per capita	300	405.8	176.8	133	1116
	*Lnpgdp*	The level of economic development	300	10.79	0.456	9.586	12.09

## 5. Empirical analysis results

### 5.1 Benchmark regression results

The benchmark regression results are shown in Table 2 below, where columns (1) and columns (2) consider the control variables and do not consider the control variables, respectively. The number of green patent grants measures the impact of Digital Inclusive Finance on green technology innovation. Columns (3) and (4) are the impact of Digital Inclusive Finance on green technology innovation as measured by the number of green patent applications when controlling variables are considered and control variables are not considered, respectively. As can be seen from the table, whether the control variables are considered or the number of green patent grants and applications are used to measure green technology innovation, the coefficient of influence of inclusive digital finance on green technology innovation has passed the test at the significance level of 1%, and the coefficient is positive. This verifies that inclusive digital finance can reduce the information asymmetry between the two sides of the credit, reduce transaction costs, and broaden the financing channels of green enterprises, thereby promoting green technology innovation and verifying hypothesis 1.

**Table 2:** Benchmark regression results.

variable	*Gtp*1		*Gtp*2	
	(1)	(2)	(3)	(4)
Digital Inclusive Finance(*Inf)*	1.932**	1.576**	2.507**	2.210**
	(6.467)	(5.217)	(7.407)	(5.940)
The level of traditional financial development(*Tf)*		0.056		0.055
		(0.703)		(0.579)
Fiscal decentralization(*Finadp)*		-0.297**		-0.308*
		(-2.404)		(-1.729)
Market-oriented index(*Mi)*		-0.006		0.050
		(-0.056)		(0.323)
The level of human capital per capita(*Hc)*		0.479**		0.192
		(2.189)		(0.629)
The level of economic development(*lnpgdp)*		-0.106		-0.213
		(-0.860)		(-1.238)
Constant term	-0.800***	-0.587***	-1.0729***	-0.781***
	(-5.562)	(-3.148)	(-6.639)	(-3.255)
Province fixed effect	control	control	control	control
Year fixed effect	control	control	control	control
Observations	300	300	300	300
Goodness of fit	0.905	0.915	0.848	0.853

The *value t* is enclosed in parentheses

* denote*p*<0.1

**denote*p*<0.05

***denote*p*<0.01。

### 5.2 Robustness test

Because the impact of finance on the real economy is lagging, green technology innovation is also cyclical in the long term. This paper chooses to verify the impact of green technology innovation after processing the first phase of digital inclusive finance lag. Considering that the digital economy in municipalities is at the top of the list, the effect of the entire sample on green technology innovation may be magnified. Therefore, this document removes the municipality for re-estimation. In addition, the explanatory variables are replaced with *Gtp*3, the ratio of the number of green invention patents granted to all patents. The results are shown in Table 3 below. The robustness test results are consistent with the benchmark regression estimates, verifying the robustness of the benchmark regression conclusions.

**Table 3:** Robustness test results.

variable	Exclude municipalities	Replace variables	Lag one phase robustness	
	*Gtp*1	*Gtp*3	*Gtp*1	*Gtp*2
	(1)	(2)	(3)	(4)
Digital Inclusive Finance(*Inf)*	1.391***	0.857***		
	(3.750)	(3.195)		
*L1*. *Inf*			1.120***	1.570***
			(3.742)	(3.490)
The level of traditional financial development(*Tf)*	-0.002	-0.417***	0.072	0.105
	(-0.024)	(-4.080)	(0.879)	(1.045)
Fiscal decentralization(*Finadp)*	-0.336***	-0.251*	-0.207	-0.226
	(-2.687)	(-2.239)	(-1.516)	(-1.053)
Market-oriented index(*Mi)*	-0.014	-0.062	0.008	0.045
	(-0.125)	(-0.561)	(0.068)	(0.254)
The level of human capital per capita(*Hc)*	0.439*	0.293*	0.507**	0.254
	(1.781)	(1.846)	(2.373)	(0.791)
The level of economic development(*lnpgdp)*	-0.187*	-0.121	-0.205	-0.359*
	(-1.698)	(-0.831)	(-1.568)	(-1.737)
Constant term	-0.423**	0.029	-0.34*	-0.415
	(-2.267)	(0.148)	(-1.676)	(-1.299)
Province fixed effect	control	control	control	control
Year fixed effect	control	control	control	control
Observations	260	300	270	270
Goodness of fit	0.898	0.852	0.929	0.860

The *value of t* is enclosed in parentheses

* denote*p*<0.1

**denote*p*<0.05

***denote*p*<0.01.

### 5.3 Endogenous testing

Although the province and time effects are controlled in the previous empirical test, it can effectively solve some endogenous problems caused by missing variables. However, due to the influence of some unobservable factors, the impact of digital finance on green technology innovation is likely to have endogenous problems. Therefore, this paper uses the instrumental variable method to deal with the endogenous problem. Later, it uses the interactive term between the spherical distance from the provincial capital city to Hangzhou and the penetration rate of mobile phones (time-dependent) as the instrumental variable IV1 of digital Inclusive Finance. First, the development of digital Inclusive Finance in different provinces is closely related to the spherical distance between the province and Hangzhou. The distance between provinces and Hangzhou will not directly affect the green technology innovation of financial services. In addition, this paper uses Huang’s [45] and Nunn & Qian’s [46] methods to construct the tool variable IV2 by using the first-order lag value of digital inclusive finance and the interaction term of Internet broadband access users.

Finally, the explanatory and control variables are treated with a first-order lag to weaken the endogenous problem caused by reverse causality to a certain extent. This paper also uses this strategy to alleviate the endogenous problem effectively. Model 1 and model 2 in Table 4 report the results of two-stage least squares estimation by iv1 and iv2, respectively. Model 3 reports the results of the one-stage lag estimation of explanatory and control variables. It can be found that the variable coefficients of digital Inclusive Finance in (1), (2), and (3) are significantly positive, indicating that after considering the endogenous problem, inclusive digital finance can still promote the increase of green technology innovation substantially.

**Table 4:** Endogenous test results.

variable	IV1		IV2		One phase behind
	*Inf*	*Gtp*1	*Inf*	*Gtp*1	*Gtp*1
	(1)	(2)	(3)	(4)	(5)
*Inf*/*L*1.*Inf*		3.1714***		6.8410***	1.022***
		(3.552)		(5.505)	(3.668)
IV1	-0.0000***				
	(-4.853)				
IV2			0.0000***		
			(6.535)		
Control variables	control	control		control	control
Constant term	0.3775***	0.0935	0.4138***	-2.0332***	-0.213
	(4.957)	(0.338)	(6.740)	(-3.630)	(-1.203)
Province fixed effect	control	control		control	control
Year fixed effect	control	control		control	control
Observations	300	300	270	270	270
Goodness of fit		0.904		0.815	0.933

The *value t* is enclosed in parentheses

* denote*p*<0.1

**denote*p*<0.05

***denote*p*<0.01。

### 5.4 Analysis of the mediation effect

To verify whether *R&D* investment plays an intermediary effect in the mechanism of Digital Inclusive Finance to promote green technology innovation, this paper constructs an intermediary effect model for testing. The intermediate affect test results are shown in Table 5. First, column (1) results in Table 5 show that the coefficient of influence of Digital Inclusive Finance on *R&D* inputs is significantly positive at a confidence level of 1%, proving that Digital Inclusive Finance is significantly positive for *R&D* Inputs has a catalytic effect. Column (2) examines the impact of Digital Inclusive Finance on green technology innovation measured by the number of green patent grants when considering *R&D* inputs. Column (3) examines the impact of Digital Inclusive Finance on green technology innovation measured by the number of green patent applications, taking into account intermediary *R&D* inputs. The results of Table 5 show that the impact of Digital Inclusive Finance on green technology innovation is still significantly positive after the inclusion of *R&*D input variables, and the *R&D* input impact coefficient is also significantly positive at a confidence level of 1%.

**Table 5:** The results of the mediation effect of R&D investment intensity.

variable	(1)	(2)	(3)
	*R&D*	Gtp1	Gtp2
Digital Inclusive Finance(*Inf)*	0.439***	1.416***	1.948***
	(3.807)	(4.616)	(5.225)
R&D investment(*R&D)*		0.365**	0.598***
		(2.321)	(3.198)
The level of traditional financial development(*Tf)*	-0.022	0.064	0.068
	(-0.442)	(0.802)	(0.720)
Fiscal decentralization(*Finadp)*	0.201***	-0.370***	-0.427**
	(3.393)	(-2.854)	(-2.250)
Market-oriented index(*Mi)*	0.090***	-0.039	-0.004
	(2.704)	(-0.374)	(-0.026)
The level of human capital per capita(*Hc)*	0.060	0.457**	0.156
	(0.758)	(2.125)	(0.532)
The level of economic development(*lnpgdp)*	-0.238***	-0.019	-0.071
	(-3.782)	(-0.178)	(-0.475)
Constant term	-0.025	-0.578***	-0.766***
	(-0.298)	(-3.040)	(-3.141)
Province fixed effect	control	control	control
Year fixed effect	control	control	control
Observations	300	300	300
Goodness of fit	0.982	0.917	0.859

The value t is enclosed in parentheses

* denote*p*<0.1

**denote*p*<0.05

***denote*p<*0.01。

In addition, after joining *the R&D* investment, the impact coefficient of inclusive digital finance has been reduced, which proves that *R&D* investment has a part of the intermediary effect in the influence mechanism of inclusive digital finance to promote green technology innovation, which is a key factor, which verifies hypothesis 2.

### 5.5 Heterogeneity testing

**i) Regional heterogeneity test.** Due to the uneven development of China’s regional economy, the impact of the digital economy on green technology innovation may be regionally heterogeneous. Therefore, this paper divides the national sample into southern and northern regions for heterogeneity analysis, and the results are shown in Table 6 below. It can be seen that in the southern and northern regions, inclusive digital finance has a role in promoting green technology innovation. However, whether it is the number of green patent grants or the number of green patent applications to measure green technology innovation, the impact coefficient of inclusive digital finance in the northern region is larger, about 27.16 and 156.35, respectively, which is greater than the 17.96 and 17.96 in the south 160.48. This may be because the industrial structure of the north is mainly heavy industry, compared with the industrial layout of high-tech enterprises in the south. The demand for green technology innovation is greater, the technology spillover effect is higher, and the promotion effect of inclusive digital finance on green technology innovation is more significant in the north [47].

**Table 6:** Regional heterogeneity tests.

variable	south	northern	south	northern
	Gtp1	Gtp1	Gtp2	Gtp2
	(1)	(2)	(3)	(4)
Digital Inclusive Finance(*Inf)*	1.352***	1.510**	2.187***	2.304***
	(2.962)	(2.487)	(3.577)	(3.796)
The level of traditional financial development(*Tf)*	0.084	0.151*	0.200	0.179*
	(0.605)	(1.742)	(1.190)	(1.847)
Fiscal decentralization(*Finadp)*	-0.636***	-0.264**	-0.842**	-0.205
	(-2.826)	(-2.049)	(-2.335)	(-1.495)
Market-oriented index(*Mi)*	-0.044	0.023	0.069	-0.074
	(-0.249)	(0.238)	(0.253)	(-0.764)
The level of human capital per capita(*Hc)*	0.188	0.616**	-0.278	0.514**
	(0.577)	(2.478)	(-0.579)	(2.424)
The level of economic development(*lnpgdp)*	0.946***	-0.114	0.898***	-0.107
	(3.819)	(-1.112)	(2.108)	(-0.918)
Constant term	-0.715***	-0.658**	-0.940**	-0.999***
	(-2.716)	(-2.406)	(-2.532)	(-3.973)
Province fixed effect	control	control	control	control
Year fixed effect	control	control	control	control
Observations	170	130	170	130
Goodness of fit	0.897	0.945	0.838	0.919

The *value of t* is enclosed in parentheses

* denote *p*<0.1

**denote *p*<0.05

***denote *p*<0.01。

**ii) The heterogeneity of inclusive digital finance in different dimensions.** To explore the heterogeneity of inclusive digital finance at various levels, this part divides the application scope of digital inclusive finance into two levels: the depth of use and the breadth of application. The regression conclusion, which examines the impact of inclusive digital finance on the effect of technological innovation, is shown in Table 7 below. The above table shows that although the digitization index’s breadth and depth of use index are significantly positive. Regardless of the impact on the number of green patents granted or the number of green patent applications, the impact coefficient on the depth of use exceeds the breadth of use. The breadth of use is the cornerstone for the application of digital financial services, and the depth of use can more effectively realize the characteristics of big data and inclusive financial services.

**Table 7:** Regression results for different dimensional benchmark models.

variable	*Gtp*1	*Gtp*1	*Gtp*2	*Gtp*2
	(1)	(2)	(3)	(4)
Breadth of use(*lnf_di)*	0.574***		0.913***	
	(6.083)		(6.357)	
Use depth(*lnf_de)*		0.844***		1.273***
		(4.085)		(4.935)
The level of traditional financial development(*Tf)*	0.095	0.084	0.098	0.086
	(1.095)	(1.047)	(1.034)	(0.930)
Fiscal decentralization(*Finadp)*	-0.270**	-0.223*	-0.269	-0.197
	(-2.114)	(-1.880)	(-1.484)	(-1.151)
Market-oriented index(*Mi)*	0.009	-0.066	0.072	-0.042
	(0.080)	(-0.602)	(0.472)	(-0.263)
The level of human capital per capita(*Hc)*	0.482**	0.576***	0.148	0.311
	(2.229)	(2.662)	(0.503)	(1.037)
The level of economic development(*lnpgdp)*	-0.263**	-0.252**	-0.419**	-0.410**
	(-2.098)	(-2.100)	(-2.378)	(-2.407)
Constant term	-0.140	-0.155	-0.212	-0.209
	(-0.999)	(-1.067)	(-1.061)	(-1.074)
Province fixed effect	control	control	control	control
Year fixed effect	control	control	control	control
Observations	300	300	300	300
Goodness of fit	0.914	0.912	0.858	0.851

Inside the parentheses is the *value of t*

* denote*p*<0.1

**denote*p*<0.05

***denote*p*<0.01。

### 5.6 Threshold effect test

This paper tests the nonlinear mechanism [48] of inclusive digital finance for green technology innovation by threshold regression. First of all, the threshold regression *Bootstrap* is used to test whether inclusive digital finance has a threshold effect and what the threshold value is, and the results are shown in Table 8 below. The results are shown in Table 8, Figs 2 and 3. It can be seen that inclusive digital finance passes the double threshold and double threshold test at the confidence level of 1%, and there is a double threshold. The threshold values of inclusive digital finance are about 0.8273 and 0.6017, respectively.

**Fig 2:** Threshold variable first round test.

**Fig 3:** Threshold variable second-round test.

**Table 8:** Results of the threshold test for digital inclusive finance.

Threshold variables	Threshold type	Threshold values	F-statistics	P-value	BS frequency	lower limit	upper limit
Digital Inclusive Finance	First threshold	0.827***	24.780	0.006	1000	0.821	0.829
	Second threshold	0.602***	27.910	0.002	1000	0.588	0.603
	Third threshold	0.538	28.620	0.596	1000	0.523	0.545

The test results with digital Inclusive Finance as the threshold variable are shown in Table 9 below. The results show that when the level of digital Inclusive Finance is at a low level (inf ≤ 0.6017), the estimated coefficient of digital Inclusive Finance is small (about 0.83). This proves that the level of digital Inclusive Finance at this stage is low, the use cost is high, and the targeted green finance business is insufficient, resulting in little promotion of digital Inclusive Finance to green technology innovation. When the level of digital Inclusive Finance is at the middle level (0.6017 < inf ≤ 0.8273), the estimation coefficient of digital inclusive finance becomes larger (about 0.96). When the level of digital inclusive finance is high (Inf > 0.8273), the estimation coefficient of digital inclusive finance is the largest (about 1.07). It shows that with the development of digital Inclusive Finance and the financial support of green policies, the use cost of digital Inclusive Finance is reduced, and information asymmetry is alleviated. It shows that with the development of digital Financial inclusion and the financial support of green policies, the use cost of digital Financial inclusion is reduced, information asymmetry is alleviated. The efficiency of financial resources allocation to green enterprises is improved, thus enhancing the effect of digital Financial inclusion on promoting green technology innovation, which verifies hypothesis 3.

**Table 9:** Threshold regression test results.

Variable name	Coef	Std.	t-value	P-value
*Inf* (*Inf≤0*.*6017*)	0.831**	0.260	3.20	0.002
*Inf* (*0*.*60179*<*Inf≤0*.*8273*)	0.959**	0.263	3.65	0.000
*Inf* (*Inf*>*0*.*8273*)	1.074**	0.262	4.09	0.000
Control variables	control	control	control	control
Province fixed effect	control	control	control	control
Year fixed effect	control	control	control	control
Constant term	0.111	0.112	0.990	0.321
Observations	300	300	300	300

The *value of t* is enclosed in parentheses

* denote*p*<0.1

**denote*p*<0.05

***denote*p*<0.01。

## 6. Conclusions and recommendations

### 6.1 Research summary

In recent years, the national government has promulgated several policies to promote further the development of digital inclusive finance, which has laid a solid foundation for China to create a good financial environment to better and faster promote the development of regional green technology innovation. This paper incorporates digitally inclusive finance, R&D investment, and regional green technology selection into the framework based on existing research. Based on summarizing the existing research results, this paper puts forward the direct, indirect, and nonlinear transmission mechanisms of digitally inclusive finance and green technology innovation. Based on the "Peking University Digital Inclusive Finance Index" and the panel data of all provinces and cities in China from 2011 to 2020 as samples, this paper uses the panel fixed effect model and threshold regression model to verify the impact and mechanism of digital inclusive finance on regional green technology innovation. It measures R&D investment by the ratio of internal expenditure on research and experimental development in each region to provincial GDP. It also measures the level of green technology innovation in various provinces (municipalities and autonomous regions) through the number of green patent grants and applications.

The benchmark regression shows that whether the number of green invention patents granted or the number of green invention patents declared to evaluate green technology innovation, digital inclusive finance has a significant positive impact on green technology innovation. This idea remains robust after the exclusion of municipal samples, the constriction of significant explanatory variables, and the replacement of explanatory variables. After considering the endogenous problem, inclusive digital finance can still substantially promote the increase of green technology innovation.

Second, inclusive digital finance has a significant positive impact on R&D investment. After joining the R&D investment, the impact coefficient of inclusive digital finance has been reduced, which proves that R&D investment has some positive intermediary effects in the impact mechanism of inclusive digital finance to promote green technology innovation.

Third, there is a heterogeneity in the impact of inclusive digital finance on green technology innovation, manifested explicitly in the stronger role of inclusive digital finance on green technology innovation in the northern region and to a higher degree. Also, compared with the breadth of application, a stronger effect on green technology innovation shows in the depth of digital inclusive finance.

Fourth, digital Financial inclusion has a threshold effect on the impact of regional green technology innovation. When the level of inclusive digital finance is greater than the second threshold value, inclusive digital finance has the greatest role in promoting the ability of green technology innovation.

### 6.2 Policy recommendations

Based on the above empirical analysis conclusions and careful consideration of the actual situation of China’s development, this paper puts forward the following suggestions:

China should develop regional digital inclusive finance to improve regional green technology innovation. This requires that regional differences be fully considered in promoting digitally inclusive finance. We should vigorously promote digital infrastructure construction in the northern region, formulate greater digital inclusive finance development strategies, and fully use its technology spillover effect to promote the development of regional green technology innovation development. All regions also need to increase policy support to ensure the construction of a digitally inclusive economic infrastructure. By formulating the development plan of digital inclusive finance, the complementary integration of traditional financial means and digital inclusive finance should be strengthened to improve the financial development environment and give full play to the supporting role of digital inclusive finance in green technology innovation.

Second, improve the efficiency of resource allocation and achieve differentiated development. The starting point for developing inclusive digital finance varies from region to region. Regions with a good foundation not only need to give full play to the advantages of digital inclusive finance in the market and resource allocation but also need to actively explore the development path of digital inclusive finance combined with their resource endowment, promote the sharing and co-construction of digital inclusive finance facilities with surrounding areas, improving the resource allocation efficiency of both regions and surrounding areas. Make full use of the differences in industrial advantages in different regions to create diversified and multi-level digital inclusive financial products for different groups, realizing the coordinated improvement of regional green technology innovation efficiency.

Finally, strengthen the investment of educational resources and cultivate talents with high digital inclusive financial literacy. Considering that the financial literacy of digital inclusive financial services is relatively low, it is urgent to teach them the financial skills they need and improve their awareness of investment risks. While introducing high-quality talents, digital financing channels are actively used to increase R&D investment in green technology innovation in enterprises and regions, reduce transaction costs, and thus promote green technology innovation.

### 6.3 Limitation & future research direction

The research topic of this paper is the impact of Digital Inclusive Finance on green technology innovation under the intermediary of R&D investment. This paper can be expanded and explored from different aspects. For example, to further develop green technology innovation for a higher-quality green economy at the macro level, the role of digital inclusive finance on the high-quality growth of the green economy must be studied. In addition, this paper discusses the relationship between financial inclusion and green technology innovation from the perspective of Digital Inclusive Finance and regional heterogeneity. Finally, follow-up related research can analyze how the development of Digital Inclusive Finance brought about by the Internet revolution affects the efficiency of green innovation in various provinces and the spillover effect of space green technology innovation.

## Supporting information

S1 Data (XLS)
